RETRACTED

# Young plasma reverses anesthesia and surgery-induced cognitive impairment in aged rats by modulating hippocampal synaptic plasticity

**DOI:** 10.3389/fnagi.2022.996223

**Published:** 2022-09-06

**Authors:** Yanan Li, Qi Zhang, Wenyu Yan, Xupeng Wang, Jiaxu Yu, Chunping Yin, Qi Zhou, Zhiyong Hou, Qiujun Wang

**Affiliations:** ^1^Department of Anesthesiology, The Third Hospital of Hebei Medical University, Shijiazhuang, Hebei, China; ^2^Department of Anesthesiology, Hebei Children’s Hospital Affiliated to Hebei Medical University, Shijiazhuang, Hebei, China; ^3^Department of Neurology, The Second Hospital of Hebei Medical University, Shijiazhuang, Hebei, China; ^4^Department of Orthopedics, The Third Hospital of Hebei Medical University, Shijiazhuang, Hebei, China; ^5^NHC Key Laboratory of Intelligent Orthopaedic Equipment, The Third Hospital of Hebei Medical University, Shijiazhuang, Hebei, China

**Keywords:** cognitive impairment, synaptic plasticity, young plasma, aged, TrkB/ERK/CREB signaling pathway

## Abstract

We investigated the protective effect of young plasma on anesthesia- and surgery-induced cognitive impairment and the potential underlying mechanism using bioinformatics, functional enrichment analysis, gene set enrichment analysis, Golgi-Cox staining, dendritic spine analysis, immunofluorescence assay, western blot analysis, and transmission electron microscopy. Furthermore, we performed behavioral assessments using the open field test, the novel object recognition test, and the Morris water maze test. We identified 1969 differentially expressed genes induced by young plasma treatment, including 800 upregulated genes and 1169 downregulated genes, highlighting several enriched biological processes (signal release from synapse, postsynaptic density and neuron to neuron synapse). Anesthesia- and surgery-induced cognitive impairment in aged rats was comparatively less severe following young plasma preinfusion. In addition, the decreased levels of synapse-related and tyrosine kinase B/extracellular signal-regulated protein kinase/cyclic adenosine monophosphate response element-binding protein (TrkB/ERK/CREB) signaling pathway-related proteins, dendritic and spine deficits, and ultrastructural changes were ameliorated in aged mice following young plasma preinfusion. Together, these findings suggest that young plasma reverses anesthesia- and surgery-induced cognitive impairment in aged rats and that the mechanism is associated with the activation of the TrkB/ERK/CREB signaling pathway and improvement in hippocampal synaptic plasticity.

## Introduction

Older adult patients who have undergone anesthesia and surgery are more likely to experienced postoperative cognitive dysfunction (POCD), which usually manifests as changes in orientation, memory, thinking, attention, and other central nervous system functions that can last for several days to years, prolong hospitalization duration, and seriously affect the quality of life of patients (Evered et al., 2018; Zhan et al., 2019). POCD is a perioperative complication that is closely associated with age (Evered et al., 2017). It has a high incidence, ranging from 20 to 79% for heart surgery (Schwarz et al., 2013) and 4.1 to 22.3% for non-heart surgery (Rappold et al., 2016), and has become a global problem affecting families and communities. Therefore, there is an urgent need to develop an effective intervention for patients to prevent POCD following anesthesia and surgery.

RETRACTED

Although the mechanism of POCD is not entirely clear, numerous studies have confirmed that central nervous inflammation (Feng et al., 2017), oxidative stress (Lin et al., 2020), apoptosis (Qin et al., 2020), and changes in hippocampal synaptic plasticity (Chen et al., 2020) are closely associated with the occurrence of POCD. The long-term change in synaptic efficacy is called synaptic plasticity, which affects hippocampal function and is the basis for information coding and storage during learning and memory formation. Synaptic plasticity disorders contribute to the pathogenesis of numerous pathological states and neurodegenerative diseases. Moreover, the regulation of synaptic plasticity has a certain therapeutic effect on neurodegenerative changes (Skaper et al., 2017) and is involved in the reconstruction of brain networks following brain injury. The relationship between synaptic plasticity and cognitive impairment has been confirmed by many studies. For example, the study by Gao et al. (2021) demonstrated that synaptic plasticity is closely related to cognitive function and that anesthesia and surgery suppress synaptic function by activating mammalian target of rapamycin (mTOR) and inhibiting hippocampal autophagy. Several researchers have proposed that the central inflammatory response in older adult patients increases following surgery, and the abnormal expression of inflammatory mediators leads to the impairment of synaptic plasticity, resulting in cognitive impairment (Chen et al., 2021). Proteomic analysis has demonstrated in a POCD rat model undergoing splenectomy under sevoflurane anesthesia that the expression of synaptic plasticity-related proteins changes (Xiao et al., 2016; Yu et al., 2019).

There has been a broad range of studies confirming that pre-infusion of plasma from young mice improves the cognitive function of aged mice by enhancing the synaptic plasticity and neurogenesis of hippocampal neurons and that injection of plasma from aged mice into young mice impairs cognitive function and destroys hippocampal synaptic plasticity and neurogenesis (Villeda et al., 2011, 2014; Middeldorp et al., 2016). However, the molecular regulation mechanism underlying the effect of young plasma on nervous system structure and cognitive function in older adults remains unclear. In addition, whether pre-infusion of plasma from young rats reverses postoperative cognitive impairment induced by surgery and anesthesia in aged rats has not been reported to date.

RETRACTED

Therefore, in this study, we aimed to determine whether young plasma reduces anesthesia- and surgery-induced cognitive impairment in aged rats and explore the underlying mechanisms to provide a reference for future clinical research.

## Materials and methods

Experimental animals were cared for and used in accordance with the Chinese Guidance for the Care and Use of Laboratory Animals. Training certificates for laboratory animal practitioners were obtained by all experimenters (Certificate Nos. 20200198, 20200199, 20200200, and 20200201). The study was conducted with every effort to minimize animal suffering and use as few animals as possible. The Animal Review Board of the Third Hospital of Hebei Medical University approved the protocols pertaining to animals (Ethical code: 2021-005-1).

### Bioinformatics analysis

We downloaded young plasma-related gene expression data (GSE75416) from the Gene Expression Omnibus database^1^ and used the R language Limma package (version 3.40.6) to analyze differences in gene expression (|logFC| < 2, *p* < 0.05). Principal component analysis were performed by R software package. A volcano map of differentially expressed genes (DEGs) was generated in R using the ggplot2 package, which was used to process the GSE75416 dataset. A cluster analysis pheatmap of DEGs was created using the R software package.

### Functional enrichment analysis

For the GSE75416 dataset, gene ontology (GO) analyses was performed. The DEGs for biological processes were created by integrating GO terms and networks using the Database for Annotation, Visualization and Integrated Discovery (DAVID) online database tools.^2^ The R linguistic environment was used to map the GO pathways of DEGs using the ggplot2 packages.

### Protein-protein interaction network construction and hub gene identification

The protein-protein interaction (PPI) networks were predicted with the STRING database (version 11.5^3^). The PPI networks of DEGs were constructed with a combined score > 0.4, and the network was visualized with Cytoscape (version 3.8.0).

### Animals and group assignment

In this study, 120 healthy male or female Sprague–Dawley rats, aged 18 months, weighing 550–650 g, were provided by the Experimental Animal Center of Hebei Medical University (Permit No. SCXK 2021-004). During the experiment, all animals were kept in a temperature-controlled room and given free access to food and water at all times. Computer-based randomization was used to divide the rats into four groups after 1 week of adaptive feeding (*n* = 30): Control (group C), Control + Young Plasma (group C + Y), POCD (group POCD), and POCD + Young Plasma group (group POCD + Y).

RETRACTED

According to the method described previously (Villeda et al., 2014), 60 3-month-old Sprague–Dawley rats, weighing 200–250 g were euthanized under deep anesthesia, and intracardiac blood was obtained. Blood was collected with Ethylene Diamine Tetraacetic Acid (EDTA), centrifuged at 1000 × *g* for 10 min, the supernatant was extracted, and the bleeding slurry was separated. The plasma was divided into 100 μL quantities and stored immediately at −80°C until needed. Before use, a Slide-A-Lyzer dialyzer (Thermo Scientific, United States) was used to dialyze plasma in phosphate-buffered saline (PBS) to remove EDTA. The plasma of young rats (100 μL) was injected into the tail vein of the aged rats for once every 3 days. Rats were injected 8 times within 24 days. A similar amount of PBS was injected into the tail veins of rats in group C (Figure 1).

**FIGURE 1:** Experimental flow chart of the study (Drawn by Figdraw platform, ID:UYRPS4e4ff). Rats were treated with a young plasma injection for 24 days, comprising eight pre-infusions, and were subjected to anesthesia and tibial fracture surgery 24 h after the final pre-infusion. After the open field test, novel object recognition test, and Morris water maze test, the rats were sacrificed for a series of tests.

### Postoperative cognitive dysfunction model

According to our previous study (Wang et al., 2021), rats in groups POCD + Y and POCD underwent tibial fracture surgery 24 h after the final young plasma infusion to establish the POCD model. Before surgery, rats were housed in separate cages with shavings at 20–22°C with an alternating 12 h day-night cycle (40–60% humidity) and access to water and food. For the induction method, rats were kept in an anesthetic box containing 7–8% sevoflurane, then placed on a warming pad (3–4% sevoflurane for anesthetic maintenance) with a temperature of 36–38°C. An incision was made on the left hind paw after shaving and disinfection, and the tibial periosteum was stripped. Following tibial osteotomy, a silk thread was inserted into the intramedullary canal, and the wound was sutured. After anesthesia, rats in groups C and C + Y received only a skin incision and suture on the left hind paw. During anesthesia and surgery, rats’ vital signs were monitored using a small animal vital signs monitor (rm300, Reward Life Technology Co., Ltd.). After the operation, the rats were transferred to another warm anesthetic box and provided with pure oxygen for 15 min. When the rats awoke, they were transferred back to their cage.

RETRACTED

### Open field test

On the 29th day after anesthesia and surgery, the open field (OFT) test was conducted to test the spontaneous locomotor activity (SLA) of aged rats to exclude the effect of anesthesia and surgery-induced SLA changes on the cognitive function test results. Rats were placed on a 50 × 50 × 37 cm open field device, comprising a plexiglass wall and black floor, for 5 min for acclimation before the test. For the test, rats were placed in the center of the open field box and allowed to move freely for 5 min. Overhead video cameras recorded the activity of the rats, and the EthoVision™ XT software (Noldus Information Technology, Wageningen, The Netherlands) was used to analyze the distance, speed, and duration of open-road travel.

### Novel object recognition test

On the 30th day after anesthesia and surgery, the novel object recognition test (NORT) was used to evaluate the cognition ability of aged rats. The NORT comprises three phases: environmental adaptation, object exposure familiarization, and novel object recognition. Rats freely explored a black 60 × 60 × 40 cm box for 5 min during the adaptation phase. Then, two identical cube objects (A and B) were placed in a symmetrical position inside the experimental box, and the rats were placed on the centerline of the two objects and allowed to explore the two objects for 10 min. The detection times of each of the two objects by the rats were recorded. One hour later, the right cube object B was removed and replaced with a new cylindrical object C, and the exploration times of objects A and C over 5 min were recorded using a video analysis system (XR-XZ301, Xinruan, Shanghai, China). During the experiment, the recognition index (recognition index = new object exploration time)/(new object exploration time + familiar object exploration time) was recorded as an index of the cognitive ability of the aged rats.

### Morris water maze test

On the 31st to 35th day after anesthesia and surgery, memory and learning abilities were evaluated using the Morris water maze (MWM) test according to our previous study (Wang et al., 2021). We used a 180-cm diameter, 50-cm high, and 32-cm deep black and transparent circular pool for the water maze, which was filled with water (24–26°C). Non-toxic black ink was added to make the water opaque, and the pool was divided into four quadrants: I, II, III, and IV. A circular platform with a diameter and height of 12 cm was positioned in the middle of quadrant IV, 2 cm below the surface of the water. Around the pool, the reference substance was maintained, as were the lights in the room. The MWM test involves a 4-day training period and a 1-day detection period. During the training period, rats were placed into the water at four different starting positions facing the wall and guided to board and remain on the platform for 15 s if they failed to do so within 120 s. The pool was cleaned daily after the training session to eliminate any smell prompts. The rats underwent four training sessions per day. The escape latency (i.e., the time from which the rats were released into the pool to boarding the platform) was measured during the detection period. The time at which the original platform area was crossed within 60 s and the total time spent in the target quadrant after the platform had been removed were recorded. The MWM test was conducted using the JLBehv-MWM system (Shanghai Ji’Liang Software Technology Co., Ltd., Shanghai, China).

RETRACTED

### Golgi-cox staining

One day after the MWM test, rats were deeply anesthetized with an intraperitoneal injection of sodium pentobarbital (60 mg/kg; *n* = 8). The left hemispheres of their brains were then collected for Golgi-cox staining using a rapid Hito Golgi-Cox staining device. Briefly, the brain was collected and rinsed with normal saline and then immersed in a solution of 1:1 volumetric ratio of Hito impregnation solution mixture of A: B for 14 days at room temperature in the dark (replaced once after 24 h of immersion). Solution-3 was used to store the brains after impregnation for 2 days at 4°C (the solution was replaced once after 12 h). The brain sample was then mounted onto a vibrating slicer fixed table and sectioned at 80 mm. After mounting the brain sections onto a chromic acid gelatin-coated glass slide, staining and further processing were performed according to manufacturer instructions, and a resinous mounting medium (cat. no. 10004160, Sinopharm Chemical Reagent Co., Ltd., Shanghai, China) was applied. The target area of the brain tissue was selected for imaging with an Eclipse Ci-L photographing microscope at 200 × and 1000 ×. We ensured consistency of the background light of each photo by filling the entire field of vision with brain tissue. Images were analyzed using the Image Pro Plus 6.0 analysis software (Media Cybernetics, CA, United States) after imaging.

### Dendritic spine analysis

The cross-sectional areas of nine dendritic spines were calculated and reported as an average of four independent measurements for the dendritic spine analysis. Light microscopy (BX63, Olympus, Tokyo, Japan) was used to capture images from the pyramidal neurons in CA1. The number and length of dendritic spines within the length range of 30–90 μm on the second or third dendritic branch on the complete neuron in the center of each 1000 × image were measured to determine the density of dendritic spines per 10 μm using the following formula: the number of dendritic spines/dendritic length × 10. The Image J 1.51k analysis software (National Institutes of Health, Bethesda, Maryland, United States) was used to draw a diagram of the cell body structure of the central neurons for each 200 × image, and the Sholl analysis plug-in was used to draw 10 concentric circles with a spacing of 10 μm, centered on the cell body, and count the number of intersections between the dendrites and concentric circles.

RETRACTED

### Ultrastructure of hippocampal neurons

One day after the MWM test, the brains of the aged rats (*n* = 8) were collected for examining hippocampal neuron ultrastructure. Approximately 1 × 1 × 3 mm hippocampal tissues were collected and fixed in 4% glutaraldehyde and 1% osmium tetroxide. Tissues were dehydrated in an ethanol solution and embedded in epoxy, before staining with uranyl acetate and lead citrate. Transmission electron microscopy (H-7500; Hitachi, Tokyo, Japan) was used to examine the hippocampal synaptic density and ultrastructure of CA1. The Image-Pro Plus 6.0 image analysis software was used to record and analyze synaptic structure-related parameters (e.g., synaptic gap width) of the CA1 region of the hippocampal tissue. Synaptic density was calculated using the following formula: Nv = 8 × E × Na/π^2^, where E is the average reciprocal length of the active zone of the postsynaptic membrane, and Na is the number of synapses per photograph/the size of the photograph.

### Western blot analysis

Total protein extraction was performed using the Whole Cell and Tissue Protein Extraction Kit, as recommended by the reagent manufacturer. The Bicinchoninic Acid Protein Assay Kit (Thermo Scientific™, Waltham, United States) was used to measure protein concentrations. One day after the MWM test, the hippocampus was separated from the brain (*n* = 7), and the proteins were separated by 10% sodium dodecyl-sulfate polyacrylamide gel electrophoresis and transferred from the gel to a polyethylene difluoride membrane. After blocking the membrane with 5% skim milk powder for 2 h, the membrane was incubated overnight with primary antibodies [Postsynaptic density protein 95 (PSD95), synapsin-I, synaptophysin (SYP), growth associated protein-43 (GAP43), BDNF receptor tyrosine kinase B (TrkB), phosphorylated TrkB (p-TrkB), extracellular signal-regulated protein kinase (ERK), phosphorylated ERK (p-ERK), cyclic AMP response element binding protein (CREB) and phosphorylated CREB (p-CREB) were purchased form Abcam, and dilution in 1:800 or 1:1000 for testing]. After cleaning, the membrane was incubated with a secondary antibody for 2 h. Finally, the ultra-sensitive chemiluminescent liquid-based FujiFilm LAS 4000 imaging analyzer (FujiFilm, Tokyo, Japan) was used for visualization, and Image J (NIH, Bethesda, MD) was used to analyze the relative intensities of individual bands.

RETRACTED

### Immunofluorescence assay

One day after the MWM test, we used a triple fluorescein-labeled method to detect rat hippocampal tissues (*n* = 7). Rat hippocampal slices were cut into 20-μm thick slices for immunofluorescence staining. The samples were blocked in PBS containing 0.3% Triton X-100 (Sigma-Aldrich, Munich, Germany) and 5% bovine serum album (Beyotime, Beijing, China) for 2 h at room temperature. The samples were then incubated with synapsin-I (Proteintech, 1:100, Cat No. 17785-1-AP), p-CREB (Cell Signaling Technology, 1:100, Cat. no. 9198S), and Neun (Proteintech, 1:100, Cat No. 26975-1-AP) overnight at 4°C. The sections were washed three times with PBS before being incubated for 1 h with a goat anti-rabbit immunoglobulin G-FITC secondary antibody (1:100, Beyotime, P0186). Finally, the sections were stained using 4’,6-diamidino-2-phenylindole (DAPI; Beyotime, P0131). The fluorescence microscopy images were then quantitatively analyzed using the Image Pro Plus 6.0 software (Media Cybernetics, Inc., Rockville, MD, United States) using a Nikon Eclipse CI fluorescence microscope.

### Statistical analysis

Statistical analysis was performed using SPSS 21.0 (SPSS, Inc., Chicago, IL, United States). Data are presented as means ± standard deviations. Tukey’s multiple comparison test was performed in addition to a one-way analysis of variance for normally distributed data. A two-way repeated-measures analysis of variance and Tukey’s *post hoc* test were used to analyze the escape latency during training. Statistical significance was indicated by a *p* < 0.05.

## Results

### Screening of differentially expressed genes

The results from bioinformatics analysis showed a total of 1969 DEGs were retrieved, among which 800 were upregulated and 1169 were downregulated. The ggplot2 package of the R software was used to construct Principal component analysis diagram (Figure 2A), the visual group DEG volcano map of the GSE75416 dataset (Figure 2B), and the R software package, pheatmap, was used to draw the cluster analysis heatmap of the DEGs (Figure 2C).

RETRACTED

**FIGURE 2:** Results of bioinformatics analysis. **(A)** Principal component analysis diagram. **(B)** Differential gene volcano map. **(C)** Heatmap of differential gene cluster analysis. **(D)** GO enrichment analysis pathways. **(E)** Interaction network diagram of Top100 DEGs.

### Results of the bioinformatics analysis

The Limma package (|logFC| < 1, *p* < 0.05) was used to obtain common DEGs, which were then subjected to GO and KEGG enrichment analyses. Using the DAVID online database tools (see text footnote 2), the level of biological processes for DEGs was analyzed by integrating the GO term and network. GO pathway maps of the DEGs were drawn using R language (Figure 2D). The GO pathway diagram revealed that signal release from synapse, postsynaptic density and neuron to neuron synapse were enriched among DEGs. The STRING database was used to construct a PPI network of the DEGs, and the results revealed 23 nodes and 36 edges (Figure 2E).

### Spontaneous locomotor activity was not affected by the surgical procedure in aged rats

The OFT was used to evaluate whether anesthesia and surgery exposure induces behavioral changes due to a decrease in SLA. Results showed that the total traveled distance (Figures 3A,B; *p* > 0.05), mean traveling speed (Figure 3C; *p* > 0.05), central area residence time (Figure 3D; *p* > 0.05), and distance in center (Figures 3A,E; *p* > 0.05) were not significantly different among the four groups, which indicated that anesthesia and surgery did not reduce the SLA of aged rats.

**FIGURE 3:** Anesthesia and surgery had no effect on the spontaneous activity of the aged rats. **(A)** Traveling trajectory in the open field. **(B)** Total distance traveled. **(C)** Mean traveling speed. **(D)** Central area residence time. **(E)** Traveling distance in the center of the open field.

### Young plasma alleviated anesthesia- and surgery-induced postoperative cognitive dysfunction in aged rats

Anesthesia and surgery exposure always damages the hippocampus, which leads to learning and memory deficits (Caza et al., 2008). Therefore, we use the NORT and the MWM test to evaluate the learning and memory abilities and cognitive function of aged rats. The flow chart of the NORT, the exploration time between objects A and B in phase II, and the exploration time between object A (familiar object) and the novel object C are shown in Figures 4A–C. There were no significant differences in exploration time between objects A and B among the four groups during the object familiarization period (*p* > 0.05). The NORT results showed that the recognition index was higher in group C + Y and lower in group POCD than that in group C; moreover, the recognition index was higher in group POCD + Y than in group POCD (Figure 4D).

RETRACTED

**FIGURE 4:** Young plasma alleviated anesthesia- and surgery-induced postoperative cognitive dysfunction (POCD) in aged rats. **(A)** Schematic of the novel object recognition test (NORT). **(B)** Exploration time to the familiar object. **(C)** Exploration time to the familiar and novel objects during the novel object recognition phase. **(D)** Recognition index. **(E)** Swimming trajectory. **(F)** Escape latency. **(G)** Times of crossing the platform. **(H)** Total times spent in the target quadrant. **(I)** Average swimming speed. Data are shown as means ± standard deviations. *p < 0.05 compared with group C, **p < 0.05 compared with group POCD (*n* = 30 per group).

The results of the MWM test revealed that the escape latency was shorter and times of crossing the platform and the total time spent in the target quadrant were higher in group C + Y than in group C. The escape latency higher and the times of crossing the platform and the total time spent in the target quadrant were lower in group POCD than in group C. However, the escape latency was shorter and times of crossing the platform and the total time spent in the target quadrant was higher in group POCD + Y than in group POCD (Figures 4E–H; *p* < 0.05). There were no significant differences in swimming speed among the four groups (Figure 4I, *p* > 0.05).

### Young plasma alleviated dendritic and spine deficits in postoperative cognitive dysfunction rats

To explore the potential mechanism of young plasma in improving postoperative cognitive function in aged rats, we explored dendritic spine density and morphological alterations. The Golgi-Cox staining images showed that the dendritic length (Figures 5A,B; *p* < 0.01), dendritic number (Figures 5A,C; *p* < 0.01), and branches (Figures 5A,D; *p* < 0.05) in the CA1 region was lower in group POCD and higher in group C + Y than in group C. However, young plasma reversed the reductions in dendritic length (Figures 5A,B; *p* = 0.012), dendritic number (Figures 5A,C; *p* = 0.021), and branches induced by POCD in group POCD + Y (Figures 5A,D; *p* = 0.009). In addition, the spine density in CA1 was lower in group POCD and higher in group C + Y than in group C (Figures 5A,E; *p* = 0.015). Young plasma reversed the reduction in spine density induced by POCD in group POCD + Y (Figures 5A,E; *p* = 0.031).

**FIGURE 5:** Young plasma alleviated dendritic and spine deficits in the hippocampus of postoperative cognitive dysfunction (POCD) rats. **(A)** Representative hippocampal Golgi-Cox staining images showing dendritic arborization in hippocampal CA1 pyramidal neurons and an intersection diagram of dendritic arborization and concentric circles in hippocampal slices. Scale bar: 400 μm and 50 μm for enlarged inserts. **(B)** Quantification of the dendritic length of hippocampal CA1 pyramidal neurons. **(C)** The number of dendrites in hippocampal CA1 pyramidal neurons. **(D)** Spine density of dendrites in hippocampal CA1 pyramidal neurons. **(E)** Quantitative analysis of the number of intersections of dendrites in hippocampal CA1 pyramidal neurons. Data are shown as means ± standard deviations. *p < 0.05 compared with group C, **p < 0.05 compared with group POCD (*n* = 8 per group).

RETRACTED

We further explored the protective effect of young plasma on synaptic plasticity in POCD rats by examining the hippocampal synaptic ultrastructure in the CA1 region. Results showed that compared with group C, the synaptic density (Figures 6A,C; *p* = 0.021) was lower and the synaptic gap width was higher (Figures 6B,D; *p* = 0.019) in group POCD, and the synaptic density (Figures 6A,C; *p* = 0.021) was higher and the synaptic gap width was lower (Figures 6B,D; *p* = 0.008) in group C + Y. Young plasma enhanced synaptic density (Figures 6A,C; *p* = 0.008) and reduced the synaptic gap width in group POCD + Y compared with group POCD (Figures 6B,D; *p* = 0.032).

**FIGURE 6:** Young plasma improved the ultrastructure of hippocampal synapses. **(A)** Representative images of hippocampal synapses under transmission electron microscope (TEM). The yellow arrows indicate synapse. Scale bar: 1 μm. **(B)** Representative images of single synapse. The position between two gray arrows indicate synaptic gap width. Scale bar: 500 nm. **(C)** Quantitative statistics of synaptic density in different groups. **(D)** Quantitative analysis of synaptic gap width. Data are shown as mean ± SD. *P < 0.05 compared with group C, **P < 0.05 compared with group POCD (*n* = 8 per group).

### Young plasma upregulated the expression of synapse-related proteins in the hippocampus of postoperative cognitive dysfunction rats

We evaluated the expression of synaptic markers in the hippocampus. The bands illustrated that the expression level of PSD95 (Figure 7A; *p* = 0.021), SYP (Figure 7B; *p* = 0.035), GAP43 (Figure 7C; *p* = 0.026), and synapsin-I (Figure 7D; *p* = 0.013) were significantly downregulated in group POCD and upregulated in group C + Y compared with group C, whereas the expression level of PSD95, SYP (Figure 7B; *p* = 0.038), GAP43 (Figure 7B; *p* = 0.029), and synapsin-I (Figure 7D; *p* = 0.016) were significantly upregulated after pre-infusion of young plasma in group POCD + Y compared with group POCD. The colocalization of Neun with synapsin-I in the CA1 region using immunostaining was conducted to confirm the results obtained from the western blot analysis. Results revealed that the abundance of synapsin-I was markedly lower in group POCD and higher in group C + Y than in group C (Figures 7E,F; *p* = 0.022), whereas the abundance of synapsin-I was higher after pre-infusion of young plasma in group POCD + Y than in group POCD (Figures 7E,F; *p* = 0.026).

RETRACTED

**FIGURE 7:** Young plasma increased the synapse-associated protein expression in postoperative cognitive dysfunction (POCD) rats. The expression of synapse-associated proteins including **(A)** PSD-95, **(B)** SYP, **(C)** GAP-43 and **(D)** synapsin-I. **(E)** Representative immunostaining showing the colocalization of Neun (green), synapsin-I (red), and DAPI (blue) in the hippocampus of CA1. Scale bar: 200 μm. **(F)** Bar graph summarizing the fluorescence intensity of synapsin-I in the hippocampal CA1. Data are shown as means ± standard deviations. *p < 0.05 compared with group C, **p < 0.05 compared with group POCD (*n* = 7 per group).

### Young plasma activated the tyrosine kinase B/extracellular signal-regulated protein kinase/cyclic adenosine monophosphate response element-binding protein signaling pathway to exert a neuroprotective effect in postoperative cognitive dysfunction rats

Previous research has demonstrated that the activation of the TrkB/ERK/CREB signaling pathway plays an important role in the improvement of synaptic plasticity via several neuroprotective measures (Tan et al., 2021). Therefore, we speculated that it also plays an important role in the alleviating effect of the pre-infusion of young plasma on POCD in aged rats. To test this hypothesis, we first evaluated the expression of coactivators (p-TrkB, p-ERK, and p-CREB) using western blot analysis. The bands showed that the expressions of p-TrkB (Figure 8A; *p* = 0.012), p-ERK (Figure 8B; *p* = 0.009), and p-CREB (Figure 8C; *p* = 0.006) were significantly downregulated in the hippocampus of rats in group POCD and upregulated in group C + Y compared with group C. The expressions of p-TrkB, p-ERK, and p-CREB were upregulated in group POCD + Y compared with group POCD. However, the expressions of TrkB, ERK, and CREB did not differ among the four groups. The dual immunostaining of Neun and p-CREB downstream of the TrkB/ERK/CREB signaling pathway revealed that the optic density of intranuclear p-CREB in the hippocampus was visibly higher in group C + Y and lower in group POCD than in group C, whereas it was higher in group POCD + Y than in group POCD (Figures 8D,E; *p* = 0.011).

**FIGURE 8:** Young plasma activated the tyrosine kinase B/extracellular signal-regulated protein kinase/cyclic adenosine monophosphate response element-binding protein (TrkB/ERK/CREB) signaling pathway to exert a neuroprotective effect in postoperative cognitive dysfunction (POCD) rats. The expression of proteins related to the TrkB/ERK/CREB signaling pathway including phosphorylated TrkB/TrkB **(A)**, phosphorylated ERK/ERK **(B),** and phosphorylated CREB (pCREB)/CREB **(C)**. **(D)** Representative immunostaining showing the colocalization of Neun (green), p-CREB (red), and DAPI (blue) in the CA1 of the hippocampus. Scale bar: 200 μm. **(E)** Bar graph summarizing the fluorescence intensity of p-CREB in the hippocampal CA1. Data are shown as means ± standard deviations. *p < 0.05 compared with group C, **p < 0.05 compared with group POCD (*n* = 7 per group).

RETRACTED

## Discussion

Our study aimed to determine the effect of young plasma on POCD in aged rats and clarify the underlying mechanisms. Our results demonstrated that young plasma improves recognition ability and attenuates learning and memory impairments in aged rats with POCD. We also found that young plasma increased the length, number, branches, and synaptic density of dendrites and decreased the synaptic gap in the CA1 region of the hippocampus of aged POCD rats. In addition, we showed that the TrkB/ERK/CREB signaling pathway plays a role in the young plasma-induced neuroprotective effect on the POCD of aged rats. Our results indicate that young plasma may serve as a potential therapeutic target for the prevention of POCD by enhancing hippocampal synaptic plasticity (Figure 9).

**FIGURE 9:** Schematic diagram of the neuroprotective effect of young plasma (Drawn by Figdraw platform, ID:WARIWa686f). Young plasma improves synaptic plasticity by activating TrkB/ERK/CREB signaling pathway, thereby inhibiting cognitive impairment caused by surgery and anesthesia.

Patients who undergo surgery often experience POCD, which is a severe postoperative neurological complication (Terrando et al., 2011; Mashour et al., 2015). Neurotoxicity has been observed in patients treated with inhalational and intravenous anesthetics (Bosnjak et al., 2016; Xu et al., 2018). Furthermore, numerous studies have demonstrated that anesthesia combined with surgery can induce the development of POCD in older adults (Evered and Silbert, 2018; Miller et al., 2018; Belrose and Noppens, 2019). However, at present, there remain few effective therapies for POCD (Kotekar et al., 2018). Our results showed that there were no significant differences in movement speed, distance, or central area residence time among the four groups; thus, anesthesia and surgery did not affect the spontaneous motor function of aged rats. We also conducted behavioral experiments (i.e., the MWM test and the NORT) to test the cognitive function of aged rats. The MWM, which evaluates spatial exploration and positional navigation, is a classical method used to examine the spatial cognition of rodents. In the NORT, rodents’ innate instincts to approach and explore novel objects are observed to evaluate recognition memory. The experimental cycle of the NORT is short, which minimizes the impact of long-term training and physical exertion on the results. Our findings revealed that sevoflurane combined with tibial fracture surgery induces postoperative cognitive impairment in aged rats, which is consistent with the results of previous studies (Zheng et al., 2017; Feng et al., 2021). Moreover, young plasma alleviated anesthesia- and surgery-induced cognitive impairment in aged rats and also improved the cognitive function of aged rats that did not undergo anesthesia and surgery, which is also in line with a previous study (Castellano et al., 2017).

RETRACTED

During the aging process, there is a reduction in certain cognitive function-related proteins, which results in the destruction of brain structure and the impairment of cognitive function (Baruch et al., 2013; Lim et al., 2013). The combination of surgery and anesthesia disrupts the hippocampal neuroinflammatory response (Subramaniyan and Terrando, 2019) and synaptic plasticity (Gao et al., 2021), and because the damage to brain tissue is greater than that during aging, the degree of cognitive function decline is greater. This explains why the incidence of POCD is higher in older adult patients than in young patients. Numerous therapeutic strategies have been developed to treat POCD, including non-pharmacological and pharmacological approaches. However, their therapeutic effects are currently inadequate because too many participants undergo non-pharmacological interventions, and there are side effects associated with the use of pharmacological approaches (Kotekar et al., 2018; Urits et al., 2019). Thus, developing more effective strategies to relieve POCD that result in fewer adverse outcomes is crucial to help older adult patients overcome POCD and reduce socioeconomic burdens.

Recently, numerous studies have reported that young plasma reduces the spontaneous cognitive function of aged rats by improving hippocampal synaptic plasticity (Gao et al., 2021; Chen et al., 2022; Xue et al., 2022). Given that the mechanism of cognitive function impairment during the aging process is similar to that following surgery and that the disruption of synaptic plasticity is also an important mechanism in the occurrence and development of postoperative cognitive impairment in older adults, we predicted that pre-infusion of young plasma would reduce the occurrence of POCD by improving hippocampal synaptic plasticity. To confirm our hypothesis, we performed bioinformatics analysis to explore the mechanism underlying the effect of young plasma on cognitive function in aged rats. Results revealed that the signal release from synapse, postsynaptic density and neuron to neuron synapse were enriched and the gene of ERK1/2 and CREB were most affected by young plasma, providing a basis for further experiments.

RETRACTED

According to the results of the bioinformatics analysis, we further examined the mechanisms underlying the beneficial effect of young plasma on POCD to determine whether young plasma may be considered a potential therapeutic target. Synaptic plasticity refers to the connection between nerve cells (i.e., a synapse), and its connection strength can be adjusted (Citri and Malenka, 2008). The synapse is a key interconnecting structure that enables information transmission between neurons and between neurons and effector cells. The structure and function of the synapse can be influenced by external stimulation or environmental factors, which are closely related to the decline in learning and memory abilities (Lisman et al., 2018). Synaptic plasticity, including long-term enhancement and inhibition, is considered the biological basis of learning and memory activities at the cellular level (Bannerman et al., 2014). Numerous studies have confirmed that anesthesia and surgical exposure can induce POCD by destroying synaptic plasticity and synaptic connections in aged rats (Xiao et al., 2018; Qiu et al., 2020; Gao et al., 2021). In this study, we performed hippocampal Golgi-Cox staining and a transmission electron microscope to detect dendritic length, number, and branches, as well as the ultrastructure of synapses in the hippocampal CA1 region. Our results showed that young plasma significantly upregulated synaptic plasticity-related proteins (synapsin-I, PSD95, SYP, and GAP43), increased synaptic length, number, branches, and density, and decreased synaptic gap width, which is consistent with the study by Castellano et al. (2017). Although anesthesia and surgery can destroy the hippocampal synaptic plasticity of POCD rats, downregulate synapsin-I, PSD95, SYP, and GAP43, decrease synaptic length, number, branches, and density, and increase synaptic gap width, these effects can be reversed by young plasma, which suggests that young plasma improves cognitive impairment caused by surgery and anesthesia in aged rats by improving synaptic plasticity.

Tyrosine kinase B (TrkB) is a specific BDNF receptor located on the membrane of nerve cells and is involved in the growth, differentiation, and maturation of nerve cells. BDNF is an important member of the nerve growth factor family and can regulate the growth and survival of the central nervous system. BDNF alongside biological activity causes the phosphorylation of TrkB after binding with TrkB and sequentially activates ERK and other signal proteins in the cytoplasm and nucleus, which causes a kinase cascade effect that activates the entire signal transmission system and enables synaptic function transmission (Leal et al., 2014). CREB is an important nuclear transcription factor and a key molecule of various signaling pathways. It plays an important role in neuronal growth, synaptic plasticity, learning and memory abilities, and injury regeneration. It is also an important downstream signal protein of the ERK pathway. P-ERK can translocate from the cytoplasm to the nucleus and regulate target gene expression by phosphorylating CREB. Our results showed that the expression of p-TrkB decreased significantly following anesthesia and surgical exposure, which is consistent with our previous study (Yin et al., 2022). In addition, studies have confirmed that the activation of the TrkB/ERK/CREB signaling pathway can alleviate dementia and cognitive decline caused by chronic cerebral ischemia by improving synaptic plasticity (Fan et al., 2016). In this study, we found that young plasma can improve synaptic plasticity by activating the TrkB/ERK/CREB pathway, which, in turn, improved the cognitive impairment caused by surgery and anesthesia.

RETRACTED

There are several limitations to this study. We only examined the neuroprotective effects and related mechanisms of plasma from 3-month-old rats on 18-month-old rats following anesthesia and we had no special requirements for the sex of rats. The neuroprotective effect of plasma from rats of other ages or special gender and effects of aged plasma on young POCD rats need to be further explored in future studies. In addition, other POCD models using aged rats, such as splenectomy and partial hepatectomy models, should be further investigated. Furthermore, we only preliminarily explored the effect of pre-infusion of young plasma on postoperative cognitive impairment and the role of synaptic plasticity in aged rats. However, further exploration of the neuroprotective mechanism of the pre-infusion of young plasma would be valuable. Finally, effect of young plasma infusion in the patients for POCD symptom amelioration needs our further exploration.

## Conclusion

Our data showed that young plasma reverses anesthesia- and surgery-induced cognitive impairment in aged rats. The potential mechanism may be related to the activation of the TrkB/ERK/CREB signaling pathway to improve hippocampal synaptic plasticity.

RETRACTED

## Data availability statement

The datasets presented in this study can be found in online repositories. The names of the repository/repositories and accession number(s) can be found in the article/supplementary material.

## Ethics statement

The animal study was reviewed and approved by the Ethics Committee of the Third Hospital of Hebei Medical University.

## Author contributions

YL: conceptualization and writing original draft. QZha: data curation and original draft review. WY and XW: data curation and formal analysis. JY, CY, and QZho: data curation and software. ZH: resources. QW: funding acquisition and original draft review. All authors contributed to the article and approved the submitted version.

## Footnotes

1
https://www.ncbi.nlm.nih.gov/gds/

2
http://david.ncifcrf.gov/

3
http://string-db.org
